RETRACTED

# Effect of the Holistic Nursing Model of Responsibility System on the Mental State of Elderly Patients with Limb Fractures Fixed by Splints in the Emergency Department

**DOI:** 10.1155/2023/1271606

**Published:** 2023-07-07

**Authors:** Shaolan Du, Yanli Hao, Yajuan Jiao

**Affiliations:** ^1^Emergency Department, Baoji Central Hospital, Baoji, Shaanxi 721008, China; ^2^Department of Ophthalmology, Affiliated Hospital of Yan'an University, Yan'an, Shaanxi 716000, China; ^3^Department of Orthopedics, Baoji Central Hospital, Baoji, Shaanxi 721008, China

## Abstract

**Objective:**

To explore the effect of the overall nursing mode of responsibility system on the psychological state of elderly patients with limb fractures fixed by splints.

**Methods:**

This study selected 150 elderly patients who received emergency treatment of a limb fracture fixed by a traditional Chinese medicine splint in our hospital from May 2018 to June 2021 as the research subjects. They were divided into a control group and an observation group, with 75 cases in each group. The control group was intervened by traditional nursing mode, and the research group was intervened by responsible overall nursing mode. The quality of nursing work was observed and compared with the nursing staff's work quality and satisfaction, patients' psychological states and satisfaction, and the risk of clinical adverse events.

**Results:**

After management, the quality of nursing work in the two groups was significantly improved. Compared with before management, the scores of basic nursing measures, nursing of critical patients, ward environment management, disinfection and isolation, rescue drugs and instruments, and nursing document management in the observation group were significantly higher than those in the control group (*P* < 0.05). After management, the work quality and satisfaction of nurses in the two groups were significantly higher than those before management. The SERVQUAL scale score and satisfaction score in the observation group were significantly higher than those in the control group (*P* < 0.05). The scores of HAMA and HAMD in the observation group were significantly lower than those in the control group (*P* < 0.05). The overall satisfaction of nursing in the observation group was 96.00%, which was significantly higher than the 80.00% in the control group (*P* < 0.05). The incidence of adverse events in the observation group was 8.00%, which was significantly lower than 17.33% in the control group (*P* < 0.05).

**Conclusion:**

Giving elderly patients with limb fracture emergencies treated with splint fixation using traditional Chinese medicine the overall nursing mode management and responsibility system can give the elderly patients comprehensive and systematic clinical nursing, increase their trust and compliance with nursing work, improve the patient's psychological state, improve clinical satisfaction, and achieve the ideal doctor-patient relationship, which is worthy of clinical application.

RETRACTED

## 1. Introduction

Limb fracture is one of the common types of orthopedics [1]. With the aging of the population and changes in bone loss, the incidence of fractures in the elderly is increasing year by year, which seriously affects the quality of life and limb function [2]. In order to promote the rapid physical rehabilitation of elderly patients with limb fractures, clinicians often provide targeted treatment and postoperative rehabilitation nursing services according to the type, degree, and course of the fracture. Among them, traditional Chinese splint fixation has the advantages of simple operation, convenient economy, and a remarkable therapeutic effect and has been widely used in clinical practice [3, 4]. However, elderly patients need long-term bed rest after fracture, and the gastrointestinal and metabolic systems are disordered, increasing the psychological pressure and physiological needs of patients. In addition, acute and chronic diseases are often associated with the slow healing of the fracture site after clinical fixation, and the recovery of joint and limb functions is not ideal, which also delays the recovery time of the disease and aggravates the degree of physical and mental trauma [5]. Traditional postoperative rehabilitation nursing modes make it difficult to meet the nursing needs of elderly patients and their families due to their general adaptability. In addition, due to the limited number of nursing staff and trivial nursing affairs, problems such as incomplete nursing work occasionally occur, which will cause secondary harm to patients and is not conducive to compliance during nursing [6, 7]. In order to carry out the humanistic care and quality nursing service project of the Ministry of Health, pay attention to the responsibility system and reform the nursing mode in terms of the breadth and depth of quality nursing service. With the overall nursing mode of responsibility system as the core and patients as the first subject, the responsibilities of nursing staff are refined, and special specialized projects are added to carry out all-round, multilevel, and whole-process scientific nursing. In addition, the implementation of flat management will promote the comfort of nursing staff, relieve the sense of fatigue, and increase the care and nursing treatment for patients. It is applied to the training and management of the whole nursing staff in the hospital, and good nursing effects are achieved. However, no literature has been found on the application of limb fractures to emergency elderly patients [8–10]. In this study, 150 emergency elderly patients with limb fractures treated by TCM splint fixation in our hospital were respectively managed by traditional rehabilitation nursing and the overall nursing mode of responsibility system, and the intervention effects of the two groups of patients were observed. The report is as follows.

RETRACTED

## 2. Materials and Methods

### 2.1. General Information

In this study, 150 elderly patients who received TCM splint fixation for limb fractures in our hospital from May 2017 to June 2021 were selected as the research subjects and were divided into a control group and an observation group by the numerical random table method. There were 46 males and 29 females in the control group, ranging in age from 38 to 65 years old, with an average age of 57.01 ± 9.42 years old, and the course of the disease was 1.18 to 13.92 days. In the observation group, there were 48 males and 27 females, aged from 39 to 67 years, with an average age of 56.41 ± 9.52 years, and the course of the disease ranged from 1.36 to 14.03 days. There were no statistically significant differences in age, gender, disease course, and other general information between the two groups (*P* > 0.05), indicating comparability. The control group adopted routine nursing mode intervention, and the observation group adopted responsibility holistic nursing mode intervention.

### 2.2. Inclusion and Exclusion Criteria

The inclusion criteria were as follows: ① in line with the diagnostic and therapeutic criteria of TCM diseases and syndromes [11] and the diagnostic criteria of limb fracture in the scientific basis of TCM bone injury [12]; ② the patient was diagnosed with limb fracture by CT, X-ray, and other imaging examinations; ③ there were obvious traumatic sites, and all fracture types were all closed; ④ the age ranges from 18 to 75 years; ⑤ no cognitive and mental disorders; ⑥ barrier-free communication, capable of completing the questionnaire independently; and ⑦ all subjects were informed of the research content and signed informed consent.

The exclusion criteria were as follows: ① complicated with functional disorders of the heart, liver, lung, and other important organs; ② no previous surgical history, malignant tumor, or infection at the fracture site; ③ with coagulation dysfunction or severe inflammation; ④ have joined or participated in other rehabilitation research work; and ⑤ finding it difficult to comply with medical advice and having poor compliance.

RETRACTED

### 2.3. Research Methods

The control group adopted the traditional rehabilitation nursing management mode, that is, after admission, patients were instructed to fill out basic information (questionnaire, etc.), deal with admission matters, and inform themselves about the precautions of traditional Chinese medicine splint fixation. After fixation, the electrocardiogram, respiratory rate, temperature, and skin status of the patients were recorded regularly. In case of emergency, timely treatment was conducted, and feedback was reported to the attending doctor. The observation group adopted the responsibility system holistic nursing mode intervention, and some orthopedic nursing staff were selected to form a special responsibility group, including 1 orthopedics deputy director nurse, 6 nurses in charge, and 9 nurses and 9 clinical nurses. Organize members of the special responsibility group to learn the professional requirements, team spirit, and significance of the holistic nursing responsibility system and establish good nursing cognition and work attitude. Specific implementation measures were as follows: ① fixed responsibility area and personnel responsibilities: according to the ward distribution and disease situation. The chief nurse, as the head of the team, is responsible for developing nursing plans, supervising the implementation of nursing staff and the quality of work, testing the depth and breadth of nursing work implementation, dealing with critical events, and arranging a new stage of nursing plan. At the same time, I also paid attention to the transfer and arrangement of team members, the examination of first-aid drugs and instruments, and the assistance of nurses and nurses. The personnel should be reasonably arranged according to the working experience, ability, and attitude of team members; one nurse and one nurse were selected as office staff, responsible for sorting out emergency documents and patient information, answering patients' or family members' questions about disease and medication, communicating with other departments in critical situations, and applying for and reporting medication and instruments of the department. In addition, comprehensive and real-time records help grasp the progress of patients' conditions, which makes it convenient to call out emergencies. Two nurses were selected as emergency personnel to pay attention to the environment, temperature, humidity, and other controls in the operating room to increase patients' compliance during treatment. Regularly disinfect and sterilize the operating room, check and replace emergency drugs and instruments, etc., to ensure the smooth operation of fixation. Two nurses were selected as bed nurses, and each nurse guaranteed 6 to 8 patients, providing basic nursing, emergency nursing, special nursing, and psychological comfort actively communicate with patients and their families, increase nurse-patient relationships, improve patient satisfaction, etc. At the same time, pay attention to the patient's physical state and record regularly to ensure the smooth development of nursing work. The nursing nurse should regularly observe the patient's consciousness, body position, skin, pupil, and temperature and make detailed electronic records. In case of an emergency, the office nurse or nurse will sort out the patient's information, past history, and matters needing attention in time. The responsible nurse should timely understand and satisfy the needs of patients, pay attention to effective communication, and provide scientific and detailed, seamless nursing services. The responsible nurse should guide the patient's rehabilitation training regularly and assist the family members with complete body massage, skin warmth, etc. Pay attention to the patient's psychological state and comfort level, guide him/her to eat food with less oil, less salt, and easy digestion, pay attention to the changes in the patient's gastrointestinal function, and alleviate the degree of gastrointestinal function injury. ② Flexible scheduling system: the deputy director of orthopedics nurse on white spot take turns on the day shift, night shift, nurse and nurses according to the actual number of patients and data statistics. Set the morning shift, middle shift, and evening shift. The morning shift is from 8:00 to 16:00, the middle shift is from 16:00 to 24:00, and the evening shift is from 24:00 to 8:00. During the shift, the two groups of nursing staff should carefully check the ward situation, explain the situation of some patients, and address any matters needing attention. During the 2∼3 weeks' shift, pay attention to the shift between the primary and secondary situations of the nursing staff's dynamic adjustment. Among them, there are responsible nurses for patients every day, and each patient is taken care of by two responsible nurses in turn. Each nurse is responsible for 6–8 patients in a given area. (3) Perfect supervision and reward and punishment system: check content 2∼3 times a week, including ward environment, patient satisfaction, recognition of nursing work, data sorting, summary, drugs, equipment, disinfection work, etc. The inspection results are reviewed by supervisors and dealt with according to the reward and punishment system. Regularly check the professional knowledge, operational skills, and psychological state of nursing staff and constantly improve the professional quality and work quality of the nursing team.

RETRACTED

### 2.4. Observation Indicators

① Comparison of orthopedic nursing work quality: according to the quality scoring standard of orthopedic nursing work of our hospital, the work quality of the two modes before and after management for 3 months was compared. There are 6 aspects in total, including basic nursing measures, critical patient nursing, ward environmental management, disinfection and isolation, rescue medicine and instruments, nursing document management, etc. ② Work quality and satisfaction of nursing staff: the modified SERVQUAL Service Quality Scale [13] was used to evaluate the service quality of nurses before and after management for 3 months. The scale has 5 dimensions, including reliability, reactivity, assurance, empathy, and tangibility, with a total of 19 items. The 5-level scoring system is adopted. The overall score is positively correlated with patient satisfaction. The Karowski (NSNS)/Miller (MMSS) satisfaction scale [14] was used to measure the job satisfaction of nurses before and after management for 3 months. The scale has eight dimensions, including benefits, scheduling, work-family balance, relationships with colleagues, networking opportunities, professional development opportunities, work recognition and recognition, control over work, and responsibility. There are 31 entries in total. Using a 5-level scoring system, from “very dissatisfied” to “very satisfied,” with high authority. ③ Comparison of psychological status: the Hamilton Anxiety Scale [15] was used to measure the anxiety degree of patients in the two groups before and after management for 3 months. There were 14 items in total. The overall score was less than 7 as no anxiety, and 7∼13 as low anxiety. 14–20 were marked as significant anxiety; ≥21 is considered extreme anxiety. The Hamilton Depression Scale [16] (HAMD) was used to measure the depression degree of 2 groups before and 3 months after management, including anxiety/somatization, body weight, cognitive impairment, day-night change, block, sleep disturbance, and despair. No depression with an overall score ≤7; 8 to 19 were classified as mild depression; 20 to 34 are classified as moderately depressed; ≥35 was classified as major depression. ④ Comparison of nursing satisfaction: patients were interviewed by using a questionnaire of satisfaction. The questionnaire included 25 items, including nursing environment, nursing staff professional work, nursing service attitude, inpatient environment, and disease awareness. The total score is 25∼100 points, with the total score <60 being dissatisfied, 60∼74 being generally satisfied, 75∼90 being relatively satisfied, and >90 being particularly satisfied. Overall nursing satisfaction = (general satisfaction + relatively satisfaction + special satisfaction) number of cases/total number of cases × 100%. ⑤ Comparison of incidence of adverse events: the incidence of adverse events in the two groups was recorded and observed during the follow-up of 3 months, including falls, bed falls, compression injuries, lost infusion tubes, wound infections, thrombosis, etc.

RETRACTED

### 2.5. Statistical Treatment

The data were processed by SPSS 24.00 statistical software. Measurement data were expressed as *X* ± *S*, and comparison between groups was performed by *t*-test. The statistical data were expressed as the number of cases (*n*) and percentage (%), and the comparison between groups was performed by *χ*^2^ test. *P* < 0.05 indicated that the difference was statistically significant.

## 3. Results

### 3.1. Comparison of General Data between the Two Groups

The results showed that there were no significant differences in gender, age, education level, disease type, and surgical experience between the observation group and the control group (*P* > 0.05), as shown in Table 1.

### 3.2. Comparison of the Quality of Orthopedic Nursing Work

The results showed that there was no significant difference between the two groups in nursing work quality before mode management (*P* > 0.05). The nursing quality of the two groups after management was significantly improved compared with that before management. The scores of basic nursing measures, critical patient nursing, ward environmental management, disinfection and isolation, rescue medicine and instruments, and nursing document management in the observation group were significantly higher than those in the control group (Figure 1). The difference was statistically significant (*P* < 0.05), as shown in Table 2.

### 3.3. Comparison of Work Quality and Satisfaction of Nursing Staff

The results showed that there was no significant difference in the quality and satisfaction of nursing staff before management between the two groups (*P* > 0.05). The work quality and satisfaction of nursing staff in the two groups after management were significantly improved compared with that before management (Figure 2). The SERVQUAL scale score and satisfaction score of the observation group were significantly higher than those of the control group, and the differences were statistically significant (*P* < 0.05) (Figure 2), as shown in Table 3.

### 3.4. Comparison of Psychological Status between the Two Groups

The results showed that there was no significant difference in psychological status score between the two groups before management (*P* > 0.05). HAMA and HAMD scores of 2 groups after management were significantly lower than those before management. HAMA and HAMD scores in the observation group were significantly lower than those in the control group (Figure 3), and the differences were statistically significant (*P* < 0.05), as shown in Table 4.

RETRACTED

### 3.5. Comparison of Clinical Nursing Satisfaction

The results showed that the overall nursing satisfaction of the observation group was 96.00%, which was significantly higher than that of the control group at 80.00% (Figure 4). The difference was statistically significant (*P* < 0.05), as shown in Table 5.

### 3.6. Comparison of Incidence of Adverse Events

The results showed that the incidence of adverse events in the observation group (8.00%) was significantly lower than that in the control group (17.33%) (Figure 5). The difference was statistically significant (*P* < 0.05), as shown in Table 6.

## 4. Discussion

In elderly patients, limb fractures can be accompanied by severe pain and other complications due to bone loss and body decline. It causes serious negative effects on patients' physiology and psychology, delays fracture healing time, increases psychological burden, and increases clinical treatment difficulty. Traditional Chinese medicine splint is often used in emergency elderly patients with limb fracture to maintain the original structure such as body diaphysis and joints. In terms of operation, the fracture healing effect is good, and the clinical treatment effect is good. Relevant studies have shown that after splint treatment for elderly fracture patients, high-quality nursing can promote patients' development of a good psychological state, improve nursing satisfaction, and reduce the risk of adverse events [17]. The traditional nursing management mode is mostly assigned according to the work content of medical staff, and there is no unified standard for nursing items and quality, which may cause psychological trauma to patients [18]. The holistic nursing mode of responsibility takes the patient as the core of nursing, rationalizes the arrangement, and refines the work flow and responsibility through the nursing staff. Establish a one-to-one or two-to-one nurse-patient relationship between patients from admission to discharge and take comprehensive and systematic nursing measures for patients. In order to promote their rapid recovery, adjust their psychological state and nursing satisfaction, and achieve high efficiency and excellent nursing quality [19]. At present, the overall nursing mode of responsibility system at home and abroad mostly emphasizes the assistance of nursing staff in multiple departments, with limited effectiveness in personnel management and limited attention to specific groups [20]. In this study, the nursing staff's professional quality and professional ability were significantly improved by adopting responsibility system holistic nursing mode management for elderly patients with limb fracture treated by TCM splint fixation. It can improve the bad mood of elderly patients, improve nursing satisfaction, reduce the risk of adverse events, and provide a basis for rehabilitation nursing of limb fractures.

RETRACTED

Quality nursing service can increase patients' trust and tolerance for disease treatment and improve their compliance with clinical work through the assistance ability, professional nursing knowledge, and level of cooperation between nursing teams. Service quality, professional level, and service attitude of nursing staff can be reflected by the SERVQUAL scale and satisfaction scale. The SERVQUAL scale comprehensively evaluates the service quality of service-oriented organizations through the appearance and feeling of service objects to service personnel, the performance of commitment, handling attitude and efficiency, professional knowledge level, and personalized service [21]. Patestos et al. [22] applied holistic nursing education to comprehensive student growth management, providing holistic and excellent holistic nursing concept for nursing staff, alleviating work fatigue and lack of empathy, devoting themselves to nursing work, and achieving significant self-growth ability. According to Wang et al. [23], in the application of TCM and acupuncture, the holistic nursing model of responsibility can promote the cooperative and positive abilities of nursing staff, provide a good healing space for patients, promote and stimulate the maximum healing ability of patients, and provide a good rehabilitation platform for their functional recovery. The results showed that the quality of nursing work in the two groups was significantly improved after management compared with before management. And the scores of basic nursing measures, critical patient care, ward environmental management, disinfection and isolation, rescue medicine and instruments, and nursing document management in the observation group were significantly increased compared with the control group. After management, the work quality and satisfaction of nursing staff in the two groups were significantly improved compared with those before management, and the SERVQUAL scale score and satisfaction score in the observation group were significantly increased compared with those in the control group. It is consistent with the research results of Patestos and Wang, indicating that the holistic nursing model of responsibility system can significantly improve the quality of department management and improve the work quality and satisfaction of nursing staff. The overall nursing mode of responsibility system can accurately implement the responsibilities and job processes of nursing staff, master professional-related skills, give full play to the work efficiency of nursing staff, increase the enthusiasm of nursing staff, increase the nurse-patient relationship and intimacy, and meet the needs of patients and their families as far as possible. In addition, a clear division of responsibilities and supervision system can accurately track patient conditions, reduce unnecessary waste of time and resources, significantly improve the sense of responsibility and job satisfaction of nursing staff, and lay the foundation for rationalizing the allocation of nursing workers. At the same time, a reasonable and flexible scheduling system can promote the nursing staff to coordinate the relationship between life, work, and family, which is beneficial to reducing the sense of empathy fatigue among nursing staff and increasing job satisfaction and self-confidence.

RETRACTED

Elderly patients need long-term bed rest after splint fixation after a fracture because limb function is limited and it is easy to produce depression, anxiety, and other bad emotions. In addition, due to the long postoperative recovery time, there will be pain and adverse events during the recovery, further increasing the psychological burden of patients and affecting the prognosis and quality of life. HAMA, HAMD scale, as one of the authoritative mental health test scales in the world, uses multiple aspects to reflect the degree of depression and anxiety, allowing people to quickly determine their own mental health state. Ding and Wang et al. [24] adopted a holistic nursing mode of intervention for patients with chronic pulmonary heart disease combined with heart failure, which can significantly improve the clinical symptoms of patients, relieve their negative emotions, increase the compliance of treatment and prognostic care, and improve their living standards. The results showed that HAMA and HAMD scores in the two groups after management were significantly lower than those before management, and HAMA and HAMD scores in the observation group were significantly lower than those in the control group. The overall nursing satisfaction of the observation group was significantly higher than that of the control group. The incidence of adverse events in the observation group was significantly lower than that in the control group. Consistent with the research results of Ding and Wang et al., it indicates that the application of holistic nursing mode of responsibility system in elderly patients with limb fracture emergencies can relieve their depression, anxiety, and other emotions; reduce the incidence of adverse events; and improve their satisfaction with nursing services. The holistic nursing model of responsibility system can pay comprehensive and systematic attention to patients' physiological and psychological changes through a clear division of responsibilities. The whole process of tracking and taking special nursing services with patients and their families is intended to establish a harmonious, kind doctor-patient relationship, increase patients' awareness of the disease and confidence, and relieve the psychological pressure on patients. Timely adjustment of rehabilitation nursing training programs and indicators reduces the risk of adverse events and improves patients' recognition of and satisfaction with nursing work.

RETRACTED

To sum up, the elderly patients with limb fractures treated with traditional Chinese medicine splint fixation emergency management system holistic nursing model. On the one hand, it can standardize the working process and operation of nursing staff, optimize their own professional skills, improve their job satisfaction, and improve their work enthusiasm. On the other hand, it can provide comprehensive, systematic, and scientific high-quality nursing services for fracture patients, improve their psychological state, reduce the incidence of adverse events, and meet their clinical nursing needs. However, the sample size of this study is limited, so it is necessary to expand the sample size to explore its universality. In addition, no systematic management mode has been formed, so unified standards and quality requirements under this mode need to be explored.

## Figures and Tables

**Figure 1:** Comparison of orthopedic nursing quality. The scores of basic nursing measures, critical patient nursing, ward environmental management, disinfection and isolation, rescue medicine and instruments, and nursing document management were compared with the two groups in nursing work quality before and after mode management.

**Figure 2:** Comparison of work quality and satisfaction of nursing staff. The SERVQUAL score and NSNS score were compared with the two groups in nursing work quality before and after mode management.

**Figure 3:** Comparison of the psychological status between the two groups. The HAMA score and HAMD score were compared with the two groups in nursing work quality before and after mode management.

**Figure 4:** Comparison of overall nursing satisfaction. The overall nursing satisfaction was compared with the two groups after mode management.

RETRACTED

**Figure 5:** Comparison of adverse events. The adverse events were compared with the two groups after mode management.

**Table 1:** Comparison of general data between the two groups.

Group	Control group (*n* = 75)	Observation group (*n* = 75)	Statistics	*P* value
Gender (example)				
Male	46 (61.33)	48 (64.00)	4.613	0.231
Female	29 (38.67)	27 (36.00)		
Average age (years)	57.01 ± 9.42	56.41 ± 9.52	3.921	0.130
Course of disease (day)	1.18∼13.92	1.36∼14.03	5.032	0.057
Fracture site (case)				
Humerus	18 (24.00)	19 (25.33)	0.195	0.104
Foot radius	24 (32.00)	25 (33.33)		
Femoral	16 (21.33)	14 (18.67)		
Tibiofibula	17 (22.67)	17 (22.67)		
Cause				
Weight crushed	21 (28.00)	26 (34.67)	6.120	0.212
Traffic accident	38 (50.67)	35 (46.67)		
High fall injury	16 (21.33)	14 (18.67)		
Education level				
Technical secondary school and below	21 (28.00)	19 (25.33)	6.234	0.068
College or bachelor degree	30 (40.00)	33 (44.00)		
Master degree or above	24 (32.00)	23 (30.67)		

**Table 2:** Comparison of orthopedic nursing quality ($\bar{x}$ ± *s*, points).

Group	Time	Control group (*n* = 75)	Observation group (*n* = 75)
Basic nursing measures	Before the management	87.02 ± 9.23	87.21 ± 9.31
	After the management	91.10 ± 7.75^*∗*^	99.82 ± 5.36^*∗*^^#^

Critical patient care	Before the management	84.57 ± 9.08	84.28 ± 9.12
	After the management	90.35 ± 7.92^*∗*^	98.30 ± 6.40^*∗*^^#^

Ward environmental management	Before the management	86.02 ± 8.61	89.46 ± 8.56
	After the management	92.37 ± 7.09^*∗*^	96.92 ± 6.10^*∗*^^#^

Disinfection isolation	Before the management	77.01 ± 8.13	77.42 ± 8.35
	After the management	86.32 ± 7.25^*∗*^	91.20 ± 6.84^*∗*^^#^

Salvage medicine apparatus	Before the management	90.03 ± 8.79	90.04 ± 8.73
	After the management	95.72 ± 7.04^*∗*^	98.31 ± 6.63^*∗*^^#^

Nursing document management	Before the management	86.90 ± 9.29	86.84 ± 9.32
	After the management	94.23 ± 7.48^*∗*^	97.93 ± 7.05^*∗*^^#^

Note. Compared with the control group before management, ^*∗*^^#^*P* < 0.05.

**Table 3:** Comparison of work quality and satisfaction of nursing staff ($\bar{x}$ ± *s*, points).

Group	Time	Control group (*n* = 75)	Observation group (*n* = 75)
SERVQUAL score	Before the management	73.02 ± 9.68	73.14 ± 9.65
	After the management	83.27 ± 8.35^*∗*^	87.92 ± 8.60^*∗*^^#^

NSNS score	Before the management	89.54 ± 10.67	89.39 ± 10.71
	After the management	97.92 ± 9.41^*∗*^	128.60 ± 8.25^*∗*^^#^

Note. Compared with the control group before management, ^*∗*^^#^*P* < 0.05.

**Table 4:** Comparison of the psychological status between the two groups ($\bar{x}$ ± *s*, points).

Group	Time	Control group (*n* = 75)	Observation group (*n* = 75)
HAMA score	Before the management	18.16 ± 3.42	18.19 ± 3.39
	After the management	15.65 ± 2.17^*∗*^	12.11 ± 1.31^*∗*^^#^

HAMD score	Before the management	22.48 ± 3.24	22.43 ± 3.27
	After the management	17.93 ± 2.06^*∗*^	15.28 ± 1.14^*∗*^^#^

Note. Compared with the control group before management, ^*∗*^^#^*P* < 0.05.

RETRACTED

**Table 5:** Comparison of overall nursing satisfaction (cases, %).

Group	Control group (*n* = 75)	Observation group (*n* = 75)	*χ* ^2^	*P* value
Especially satisfied	29 (38.67)	46 (61.33)	—	—
Quite satisfied	18 (24.00)	19 (25.33)	—	—
Generally satisfied	13 (17.33)	7 (9.33)	—	—
Not satisfied	15 (20.00)	3 (4.00)	—	—
Overall nursing satisfaction	80.00%	96.00%	4.319	0.032

**Table 6:** Comparison of adverse events (cases, %).

Group	Control group (*n* = 75)	Observation group (*n* = 75)	*χ* ^2^	*P* value
Fall	6 (8.00)	3 (4.00)	—	—
Drop from bed	2 (2.67)	1 (1.33)	—	—
Compression injury	1 (1.33)	0 (0.00)	—	—
Infusion tube fell off	0 (0.00)	1 (1.33)	—	—
Wound infection	3 (4.00)	1 (1.33)	—	—
Blood clots	1 (1.33)	0 (0.00)	—	—
Incidence of adverse reactions	17.33%	8.00%	4.160	0.000

## Data Availability

The data used to support the findings of this study are available from the corresponding author upon request.
